This article has been retracted.

# Clinical Value and Imaging Features of Bedside High-Frequency Ultrasound Imaging in the Diagnosis of Neonatal Pneumonia

**DOI:** 10.1155/2022/4805300

**Published:** 2022-06-23

**Authors:** Jianchang Zhu, Peng Chen, Dazhi Jiang

**Affiliations:** Ultrasonic Center, Huaibei Maternal and Child Health Hospital, Huaibei, Anhui 235000, China

## Abstract

The aim is to solve the problem of the urgent need of a nonradiation, noninvasive, and simple-to-operate diagnostic method for neonatal pneumonia that can indicate the severity of the disease and dynamically monitor the outcome of the disease. The authors propose a bedside high-frequency ultrasound technique based on methods for evaluation in the detection and treatment of neonatal pneumonia. The results obtained are as follows: the sensitivity of neonatal lung ultrasound in the diagnosis of neonatal pneumonia was 96.6%, the specificity was 93.3%, the positive predictive value was 93.5%, and the negative predictive value was 96.5%. The sensitivity of chest X-ray in the diagnosis of neonatal pneumonia was 93.3%. Compared with the lung ultrasound and chest X-ray in the diagnosis of neonatal pneumonia, the two had a good correlation. The neonatal respiratory score was positively correlated with the lung ultrasound score, and the higher the lung ultrasound score, the more severe the disease. The score decreased by 35% after 3 days of treatment and 68% after 7 days of treatment, indicating that the lung high-frequency ultrasound score can be very effective in characterizing the treatment situation. It has been demonstrated that the lung ultrasound can be used as an imaging method for the diagnosis of neonatal pneumonia. The higher the lung ultrasound score, the more severe the disease, and the lung ultrasound score was positively correlated with the disease severity. With dynamic monitoring of the lung ultrasound and the gradual improvement of clinical symptoms after treatment, the lung ultrasound score gradually decreased; therefore, the lung ultrasound can be used for re-examination of neonatal pneumonia to evaluate the treatment effect and guidance.

## 1. Introduction

Neonatal respiratory distress syndrome (RDS) is mainly due to the lack of alveolar surfactant (PS), a series of clinical syndromes that lead to dyspnea shortly after birth and progressive aggravation. The main pathological changes are atelectasis and hyaline membrane formation, the disease is most severe within 24–48 hours after birth, it is common in dry-born infants, and the younger the gestational age, the higher the incidence. Early diagnosis, correct assessment of disease severity, early treatment, and monitoring of treatment effects can avoid unnecessary mechanical ventilation, in order to reduce the occurrence of complications such as bronchopulmonary dysplasia; reduce the mortality rate; and improve the prognosis. It is the key to the treatment of this disease. At present, the clinical diagnosis of RDS mainly relies on clinical manifestations, blood gas analysis, and chest X-ray. Not only RDS, X-ray or CT examination is required for the diagnosis of many respiratory diseases in infants and young children. X-rays require exposure to ionizing radiation, which can cause genetic mutations, damage to the gonads, and chromosomal changes that can be passed on to the next generation. Research shows that infants and young children are more sensitive to the carcinogenic effects of ionizing radiation than adults. The younger the age, the greater the harm of ionizing radiation under the same dose of ionizing radiation. Clinically, especially critically ill children often require multiple examinations to monitor the treatment effect and outcome of the disease, and as the cumulative radiation dose increases, compared with a single dose of radiation, the canceration rate is greatly increased, and the neonatal body is in the stage of rapid development. Studies have shown that cells in the differentiated phase are more sensitive to ionizing radiation, and neonatal exposure to ionizing radiation should be avoided as much as possible [1]. Severely ill neonates should not be moved, and repeatedly moving neonates increases the chance of infection and may aggravate the condition. There is an urgent need for a nonradiation, noninvasive, and easy-to-operate diagnostic method that can indicate the severity of the disease and dynamically monitor the outcome of the disease.

Clinically, pneumonia is a common neonatal disease and one of the diseases with a high mortality rate. The main clinical manifestations are shortness of breath, fever, and three concave signs. Because neonatal organs are not fully developed and do not have a relatively complete immune system, their resistance to infection is extremely low, which in turn makes neonates more prone to pneumonia. Therefore, the early diagnosis of neonatal pneumonia is particularly important, and the current diagnosis is mainly based on the patient's medical history, clinical manifestations of laboratory indicators, and chest X-ray examination. However, the diagnostic effect is poor and lacks specificity, although lung CT is the gold standard of imaging examination for neonates; CT scans have high radioactivity, so they are not suitable for neonatal examinations. Ultrasound is the most commonly used the imaging method in clinical practice (Figure 1), and the principle of ultrasound imaging is the reflection and scattering of ultrasound beams at the interface between different media. However, a high-impedance interface is formed between the gas in the lungs and the soft tissue, and the ultrasonic wave is attenuated and the tissue structure behind the interface cannot be displayed. Lung disease was previously thought to be undiagnosable by ultrasound [2]. However, with the upgradation of ultrasonic instruments and the improvement of sonographers' skills and knowledge, more and more studies have been conducted on the diagnosis of lung diseases by ultrasonics. In recent years, people have gradually learned that when the lung is injured, the amount of gas and fluid in the lung changes, which can produce some ultrasound images and artifacts. As early as the 1890s in Belgium, scholars began to try to use ultrasound to diagnose RDS. In 2012, experts from the International Federation of Ultrasound reached an international consensus on the ultrasound diagnosis of lung diseases based on evidence-based medicine. The consensus holds that the lung ultrasound is more accurate and sensitive than X-ray in diagnosing pneumothorax and pleural effusion. In recent years, with the application of lung ultrasound, bedsides high-frequency ultrasound technology has been applied to the diagnosis of neonatal pneumonia and some progress has been made, there are few related reports. To this end, the authors performed bedside high-frequency ultrasound examinations for children with neonatal pneumonia and compared them with X-ray examinations in order to explore the clinical value and imaging characteristics of bedside high-frequency ultrasound in the diagnosis of neonatal pneumonia and to provide reference data for clinical treatment and research.

At present, lung ultrasound has been used in some neonatal intensive care units to diagnose lung diseases. With the improvement of lung ultrasound technology and the proof of clinical practice, it is believed that more and more neonatal departments will use lung ultrasound to diagnose neonatal lung diseases and can reduce the radiation received by neonates. In the future, lung ultrasound may become one of the diagnostic criteria. The use of lung ultrasound equipment is relatively simple, clinicians can learn to operate in a short period of time and can be used as a bedside technology to monitor the condition and treatment effect of children any time, and it can not only diagnose neonatal diseases but also evaluate the severity of the disease and the effect of treatment, which is of great significance for the diagnosis and severity assessment of lung diseases in the neonatal intensive care unit. The lung parenchyma score not only is used to diagnose neonatal lung diseases but also has significance for the pulmonary artery spectrum in the diagnosis and treatment of lung diseases. At present, there are few studies in this area, and further research is needed [3]. In conclusion, lung ultrasound is of great significance in the diagnosis and treatment of neonatal respiratory distress syndrome; it can be repeated multiple times and can dynamically monitor the treatment effect and outcome of neonatal respiratory distress syndrome. Lung ultrasound can reduce radiation exposure of children and medical staff; is fast, noninvasive, low cost, easy to operate, and can be performed at the bedside, and it is of great significance for comprehensive early diagnosis, differential diagnosis, and severity assessment of neonatal respiratory distress. In conclusion, lung ultrasound can be used as one of the routine imaging methods for the diagnosis of neonatal respiratory distress syndrome and has good specificity and sensitivity.

The authors aim to understand the accuracy, specificity, and sensitivity of lung ultrasound in the diagnosis of neonatal pneumonia; to provide another imaging method for the diagnosis of neonatal pneumonia; and to explore the 6 zones of both the lungs, the correlation between the lung ultrasound scoring method with a total score of 18 points and the severity of the disease, dynamic monitoring of the prognosis of the disease, and providing guidance for clinical diagnosis and treatment.

## 2. Literature Review

Weng et al. believe that ultrasound is an important bedside technology in emergency medicine, and clinicians can use ultrasound instruments to check and obtain results by themselves, which can make early diagnosis and timely treatment, which is of great value for the diagnosis and treatment of critically ill patients. Lung ultrasound has been used in the diagnosis of adult lung diseases, and the lung ultrasound score can assess the ventilation function and oxygenation status of the adult lungs [4]. Kim et al. suggested that compared with adults, neonatal adipose tissue, small lung volume, and thin muscle layer are more conducive to the diagnosis of lung diseases such as RDS, TTN, MAS, and neonatal pneumonia by lung ultrasound. Lung ultrasound has the advantages of simple operation, low price, bedside examination, monitoring of disease changes any time, and easy dynamic observation [5]. Severely ill neonates undergo bedside chest X-ray examination, and other neonates and medical staff in the same ward will be exposed to ionizing radiation; lung ultrasound can prevent others from being exposed to ionizing radiation. Lung ultrasound can diagnose lung disease in a timely manner and reduce the movement of the examinee. Bushnell et al. believed that it was previously thought that ultrasound could not be used for the examination of lung diseases because the lungs were filled with gas and the ultrasound was greatly attenuated by the gas and could not show the structure of the lungs, but it is gradually understood that when the lung tissue is damaged, the amount of gas in the lung decreases, the inflammatory exudate increases, changes in alveolar and interstitial air and water content can produce some ultrasound images and artifacts, the minimum resolution of ultrasound is about 1 mm, and the sensitivity to lesions is also higher [6]. Balodhi et al. studied that the pleural line can be seen in the lung ultrasound image of healthy people, that is, the linear hyperechoic under the rib and the pectoral mold line can be seen to move with the breathing movement under real-time ultrasound. Originating from the breast mold line, a series of parallel lines that are parallel to and equally spaced from the breast mold line are called A-lines. One of the abnormal lung ultrasound images is B-line, which originates from the pectoral mold line, which is perpendicular to the pectoral mold line and can radiate to the edge of the screen. In linear hyperechoic, as the air content in the lung decreases, the number of B-lines increases, and when the B-lines increase to a certain extent, lung ultrasound shows a hypoechoic area called lung consolidation. Lung ultrasound scoring methods can be used to semiquantify the severity of lung disease [7]. Wang et al. concluded that lung ultrasound has been used to diagnose various types of pneumonia in adults. Ultrasound scoring can also be used to assess the ventilation function and oxygenation status of the adult lung. Compared with adults, neonates have less adipose tissue, small lung volume, and thin muscle layer, which are more conducive to the diagnosis of neonatal lung diseases by lung ultrasound [8].

Qi et al. believed that the main treatment methods for RDS are conventional comprehensive treatment, pulmonary surfactant, and mechanical ventilation, and during mechanical ventilation, there is barotrauma and shear injury, which may lead to ventilator-related lung injury. In recent years, it has been found that, during mechanical ventilation, giving lung protection ventilation strategies can reduce ventilator-related lung injury, improve oxygenation, and improve lung compliance, including low tidal volume ventilation and lung recruitment strategies [9]. Njs et al. believed that the strategy of lung recruitment is to give an appropriate pressure within a limited time, inflate as many collapsed alveoli as possible, and at the same time, keep the open alveoli open. After lung recruitment, to keep the alveoli open to reduce shear injury, an appropriate PEEP should be given [10]. Aleem et al. believed that the evaluation of lung recruitment effect mainly relies on the oxygenation index, lung CT, and P-V curve, and the selection of the best PEEP mainly depends on the oxygenation index. Lung ultrasound score and oxygenation index were consistent in guiding the selection of optimal PEEP. Lung ultrasound scores can be used to monitor the effect of lung recruitment and select the best PEEP [11].

Khaleghnia et al. believe that although many studies in recent years have shown the advantages of lung ultrasound in diagnosing and monitoring neonatal lung diseases, the accuracy is also high, but ultrasound diagnosis of neonatal respiratory distress syndrome also has certain limitations: (1) lung ultrasound diagnosis is highly subjective, and if the operator lacks training or experience, it is difficult to ensure the accuracy of the diagnosis results, and the operator needs to undergo formal training; (2) subcutaneous emphysema will affect the performance of the ultrasound, and the lung ultrasound cannot be conducted for the diagnosis of emphysema; (3) the thicker fat layer in obese children will affect the quality of ultrasound images [12].

## 3. Research Methods

### 3.1. Research Objects

Thirty patients who were diagnosed with neonatal pneumonia in the neonatal department of a hospital from January to April 2021 were selected as the observation group, and 30 neonates without lung disease who were admitted to the hospital during the same period were selected as the control group, including 31 males and 29 females .

The clinical data of the observation group and the control group are shown in Table 1, and there were no significant difference in the clinical data (*P* > 0.05) [13].

According to the diagnostic criteria of severe pneumonia in “Zhu Futang Practical Pediatrics”:

1. Obvious symptoms of systemic poisoning
2. Shortness of breath, cyanosis, obvious dyspnea, blood gas analysis indicates respiratory failure, and ventilator-assisted ventilation treatment is required
3. The chest X-ray shows that multiple lung lobes are damaged or the extent of lung infiltration is greater than 2/3 of the lungs [14]
4. Other systems are seriously affected; severe pneumonia is defined as meeting more than one of the above criteria, divided into severe group of 12 cases and mild group of 18 cases

The clinical data of the severe group and the mild group are shown in Table 2, and there were no statistical difference in the clinical data (*P* > 0.05):

  Observation group: met the diagnostic criteria for neonatal pneumonia, and the diagnostic criteria are (1) having clinical symptoms such as fever, shortness of breath, cyanosis, apnea, cough, spit, or moaning; (2) dry and wet rales could be heard on auscultation of both lungs; (3) the chest X-ray showed thickening of lung markings, decreased permeability, punctate or patchy shadows of different sizes, consolidation shadows, etc.; (4) laboratory examination of white blood cells can be normal, increased or decreased, CRP can be increased, and blood gas analysis suggests carbon dioxide retention or hypoxemia [15]
  Control group: admitted to the hospital with other systemic diseases during the same period, no lung disease, and no clinical symptoms of pneumonia

### 3.2. Examination and Treatment Methods

#### 3.2.1. Ultrasound Examination

In a quiet state, the child was examined in the supine position, and the midsternal line, the line connecting the double nipples, the anterior axillary line, and the posterior axillary line were used as boundaries, and each lung of the newborn was divided into three parts (upper left, lower left, left axilla, upper right, right lower, and right axilla); lung ultrasound scoring was performed by scanning each lung region laterally and longitudinally with an ultrasound linear probe. Children in the observation group and control group underwent lung ultrasonography immediately after admission [16].

#### 3.2.2. Scoring Method

Each area was scored separately, with 0, 1, 2, and 3 points, with a full-score of 18 points; only A-line is displayed as 0 points, and scattered B-lines (more than 3) were scored as 1 point, massive or fused B-lines with or without subpleural consolidation were scored as 2 points, extensive lung consolidation was scored as 3 points, and the ultrasound scores for each area were summed up for the total score.

There are various methods for the division of lung ultrasonography in China; among them, the 12-zone double lung method is mostly used, that is, each side of the lung is divided into 6 areas: anterior-upper, anterior-lower, axillary-upper, axillary-lower posterior-upper, and posterior-lower. The author adopted Brat *R*'s scoring method of 6 areas of both lungs mainly because if it is divided into front and rear areas for scoring, it will lead to the overlap of inspection areas and affect the inspection results. Neonatal patients with severe pneumonia should avoid moving and stimulating them as much as possible; in order to prevent the tracheal intubation from falling off and aggravating the disease, the method for the 6-zone bilateral lung is simpler to operate, does not need to move the patient, takes less time, and can get the results quickly [17].

#### 3.2.3. Chest X-Ray

The chest X-ray examination should be completed within 24 hours after admission, and the child who is standing or unable to move can take the chest X-ray in the supine position for diagnosis by a professional radiologist.

#### 3.2.4. Clinical Observation Indicators

1. Respiratory score of neonates: on admission, the neonatal respiratory status was scored from respiratory rate, inspired oxygen concentration, moaning, three concave signs, lung auscultation, and gestational age; the higher the score, the more severe the dyspnea [18]. The children were scored immediately after admission, and the scoring criteria are shown in Tables 3 and 4.
2. Lung ultrasound imaging manifestations of neonatal pneumonia.
3. Comparison of lung ultrasound and chest X-ray in the diagnosis of neonatal pneumonia.
4. Observation of the relationship between the lung ultrasound score and the severity of neonatal pneumonia.
5. Dynamic monitoring of lung ultrasound imaging changes.
6. Recording the clinical symptoms and pulmonary signs of the neonates in the observation group such as fever, shortness of breath, cyanosis, apnea, coughing, spit, or moaning, and recording the white blood cell count and laboratory test results such as CRP [19, 20].

## 4. Analysis of Results

### 4.1. Ultrasound Imaging Results of Neonatal Pneumonia

From the above, in this experiment, the neonatal pneumonia cases involved were confirmed to have pneumonia symptoms after ultrasound examination [21, 22].

### 4.2. Diagnosis of Neonatal Pneumonia by High-Frequency Ultrasound

It can be seen from Table 5 that the sensitivity of high-frequency ultrasound for the diagnosis of neonatal pneumonia was 96.6%, the specificity was 93.3%, the accuracy was 95%, the positive predictive value was 93.5%, and the negative predictive value was 96.5% [23].

### 4.3. Comparison of Diagnostic Results between High-Frequency Lung Ultrasonography and Chest X-Ray

Among the 30 cases of neonatal pneumonia, 28 cases had pneumonia changes on chest X-ray, and 2 cases had no pneumonia changes; the sensitivity of chest X-ray in diagnosing pneumonia was 93.3%.

As it can be seen from Table 6, high-frequency lung ultrasonography and chest X-ray showed good agreement [24].

### 4.4. Correlation Analysis of Lung High-Frequency Ultrasound Score and Neonatal Respiratory Score

As it can be seen from Figure 2, *r* = 0.957 and *P* < 0.001, indicating that the score of high-frequency lung ultrasound is positively correlated with the neonatal respiratory score [25].

## 5. Conclusion

Bedside high-frequency ultrasound can be operated at the bedside of the child, which can better monitor the condition of the child in real time, can reflect the dynamic characteristics, and can obtain information in a short period of time to avoid strong ionizing radiation to the newborn. However, X-ray cannot be monitored in real time, and bedside high-frequency ultrasound just makes up for the insufficiency of X-ray. However, the operation of high-frequency ultrasound needs to be performed by experienced physicians. In addition, ultrasound also has certain difficulties in diagnosing lesions located in the center of the lung, which should be the limitation of ultrasound. Lung ultrasound can be used as an imaging modality for the diagnosis of neonatal pneumonia. The higher the lung ultrasound score, the more severe the disease, and the lung ultrasound score was positively correlated with the disease severity. From the dynamic monitoring of the lung ultrasound, with the gradual improvement of clinical symptoms after treatment, the lung ultrasound score gradually decreased, so the lung ultrasound can be used for the review of neonatal pneumonia to evaluate the treatment effect and guidance.

## Figures and Tables

**Figure 1:** Ultrasound imaging technology.

**Figure 2:** Correlation analysis of lung high-frequency ultrasound score and neonatal respiratory score.

**Table 1:** Comparison of data between the observation group and the control group.

Grouping	Gestational age	Weight	Age
Observation group	32.6 ± 5.5	3.1 ± 1.7	12.8 ± 8.2
Control group	35.2 ± 3.6	3.3 ± 1.2	11.3 ± 15.1
*t*	1.671	1.45	1.56
*P*	*P* > 0.05	*P* > 0.05	*P* > 0.05

**Table 2:** Comparison of data between the severe group and the mild group.

Grouping	Gestational age	Weight	Age
Severe group	34.2 ± 4.7	2.4 ± 1.3	10.5 ± 8.5
Mild group	36.5 ± 3.0	3.5 ± 0.7	11.1 ± 17.3
*t*	1.659	1.63	1.66
*P*	*P* > 0.05	*P* > 0.05	*P* > 0.05

**Table 3:** Neonatal respiratory score.

Index	Measured value	Score
Respiratory rate (times/min)	40–60	0 marks
	60–80	1 point
	≥80	2 minutes

Inhaled oxygen concentration	0.21	0 marks
	≤0.5	1 point
	>0.5	2 minutes

Moan	—	0 marks
	Stimulated	1 point
	When it is quiet	2 minutes

Three concave signs	None	0 marks
	Mild-moderate	1 point
	Severe	2 minutes

Lung breath sounds	Easy to smell	0 marks
	Reduce	1 point
	Almost none	2 minutes

Gestational age	≥34	0 marks
	30–34	1 point
	<30	2 minutes

**Table 4:** Ultrasound signs of neonatal pneumonia.

Lung ultrasound signs	Number of cases
Abnormal breast mold line	29
A line disappears	31
Alveolar interstitial syndrome	28
Lung consolidation	18
Lung pulsation	5
Lung slip disappeared	5
Pleural effusion	2

**Table 5:** Diagnosis results of neonatal pneumonia by high-frequency lung ultrasound.

Lung ultrasound	Gold standard		Total
	Pneumonia	Nonpneumonia	
Pneumonia	29	2	31
Nonpneumonia	1	28	29
Total	30	30	60

**Table 6:** Diagnostic results of high-frequency lung ultrasonography and chest X-ray.

Lung ultrasound	Chest radiograph		Total
	Pneumonia	Nonpneumonia	
Pneumonia	28	1	29
Nonpneumonia	0	1	1
Total	28	2	30

## Data Availability

The data used to support the findings of this study are available from the corresponding author upon request.
